# PathogenDx Detect^X^ Combined Demonstrates Equivalent Performance in Comparison to Four AOAC Certified Methods for the Detection of *Aspergillus* Species, *Salmonella* Species, and STEC in Dried Hemp Flower

**DOI:** 10.1093/jaoacint/qsad027

**Published:** 2023-02-23

**Authors:** Benjamin A Katchman, Michael Tomchaney, Austin Rueda, Shaun Stice, Mike Hogan

**Affiliations:** PathogenDx, Inc., Tucson, AZ 85719, USA; PathogenDx, Inc., Tucson, AZ 85719, USA; PathogenDx, Inc., Tucson, AZ 85719, USA; PathogenDx, Inc., Tucson, AZ 85719, USA; PathogenDx, Inc., Tucson, AZ 85719, USA

## Abstract

**Background:**

The PathogenDx Detect^X^ Combined method is a certified *Performance Tested Method*^SM^ (012201) that is enrichment-free and utilizes a DNA microarray-based end point PCR method for the simultaneous detection of *Aspergillus* (*A. flavus, A. fumigatus, A. niger, and A. terreus), Salmonella* spp., and a broad range of Shiga toxin-producing *Esherichia coli* (STEC) from hemp and cannabis flower, edibles, and concentrates.

**Objective:**

This study aimed to compare the PathogenDx Detect^X^ Combined enrichment-free method to four AOAC INTERNATIONAL certified molecular methods that utilize enrichment prior to quantitative PCR (qPCR) amplification in hemp flower for the detection of *Aspergillus (A. flavus), S. enterica,* and *Escherichia coli* 026.

**Methods:**

In this method comparison study, each method was evaluated according to the AOAC validated instructions for use (IFU) and the AOAC Appendix J validation guidelines. A total of 16 samples at three levels of contamination (0, 0.7, and 2 CFU/10g test portion) were analyzed by each method. The results for all methods were evaluated by using the probability of detection statistical model (POD).

**Results:**

Results of the validation study demonstrate that the PathogenDx Detect^X^ Combined enrichment-free method is equivalent in performance to the three proprietary methods evaluated in this study.

**Conclusion:**

The method comparison study indicated that the PathogenDx Detect^X^ Combined enrichment-free method provides equivalent detection of the target analytes (*A. flavus, Salmonella,* and a broad range of STEC) in hemp flower.

**Highlights:**

The performance of The PathogenDx Detect^X^ Combined method is significantly faster and possesses a higher or equivalent degree of sensitivity and specificity. Implementation of this method for routine microbial pathogen analysis in laboratories would save significant time and resources.

Cannabis is associated with various types of microbes that have been shown to harm immunocompromised patients (1). Metagenomic studies on cannbis plants have shown that cannabis is associated with a wide range of epiphytic and endophytic microbial communitities including several toxigenic bacterial and fungal species (2). In addition, previous studies have identified several fungal organisms in dispensary-produced cannabis, including *Aspergillus* spp. (*A. terreus*, *A. Niger*, and *A. flavus*), which is known to produce aflotoxins (2–4). State and federal regulations for cannabis safety testing reflect these findings, requiring the assessment of *Aspergillus* spp. (*A. niger, A. flavus, A. terreus, and A. fumigatus*), *Salmonella* spp., and pathogenic *Escherichia coli* (*E. coli*) in the majority of states that have legaized cannabis, with increasing safety regulations anticipated.

Traditional enrichment techniques, utilized broadly in cannabis and food safety, greatly underestimate the diversity and quantity of bacterial and fungal pathogens present in samples (5–7). While enrichment is used to increase the probability of detection (POD) of a particular pathogen, the technique is inherently flawed. Utilizing broad or selective enrichment medias introduces numerous factors including competition for nutrients, differences in relative growth rates, growth inhibitors, and the presence of bacteriophages (8–10). Enrichment therefore results in a biased, and often unpredictable, sample making it difficult to rely on specific enrichment methods as the best diagnostic approach for food and environmental safety (8–10). Molecular techniques that do not rely on in vitro growth for bacterial or fungal detection provide a more accurate representation of the pathogens, both for the diversity and quantity of the organisms present on a sample (11,12).

The PathogenDx Detect^x^ Combined method is AOAC INTERNATIONAL *Performance Tested Method*^SM^ (PTM) certified (012201) for hemp (containing <0.3% Tetrahydrocannabinol (THC)), cannabis flower, edibles (chocolates and gummies), as well as concentrates containing >0.3% THC and does not require cultural enrichment. It consists of sample DNA amplification via tandem PCR on a crude lysate, which avoids DNA purification. The Cyanine3 (Cy3)-labeled PCR product is used without amplicon cleanup, quantitation, or normalization prior to hybridization. The Cy3-labeled tandem PCR product is diluted in hybridization buffer and hybridized to the DNA microarray. The hybridized and washed microarray is then imaged to yield a Cy3 hybridization pattern distributed among the probe spots. The PathogenDx software analysis tool, Augury^©^, automatically finds the hybridized spots in the image and then calculates the median Cy3 intensity of each hybridized spot.

In this study, four different enrichment-based detection methods were evaluated and compared to the PathogenDx Detect^X^ Combined assay for the detection of *Aspergillus* spp., *Salmonella* spp., and Shiga toxin-producing *Esherichia coli* (STEC) from dried hemp flower following an unpaired study design. A total of 16 samples at three different contamination levels were evaluated with each assay. The three contamination levels consisted of: 3 samples replicate at 0 CFU/test portion, 10 replicates at 0.7 CFU/test portion (with a target of 3–7 positive samples), and 3 sample replicates at 2 CFU/test portion. All samples were enriched and analyzed according to the manufacturers’ instructions for use (IFU) for each assay as outlined in Table 1. Regardless of presumptive results, all samples were confirmed utilizing an Food and Drug Administration Bacteriological Analytical Manual (FDA BAM) methodology for that pathogen. Final confirmation was obtained by Bruker MALDI Biotyper following AOAC *Official Method of Analysis*^SM^ (OMA) **2017.09** (13).

**Table 1.** Method comparison study design: the PathogenDx Detect^X^ Combined assay was compared against four AOAC certified methods for the detection of *A. flavus*, *S. enterica*, and *E. coli* (STEC)

Matrix	Inoculating organisms^a^	Method	Contamination levels	Replicates	Test portion	Storage conditions	Enrichment
Dried hemp flower	*A. flavus* ATCC 16883 *S. enterica Enteritidis* ATCC 13076 *E. coli* 026 ATCC BAA-1653 (lyophilized)	PathogenDx Detect^X^ Combined	0 CFU/test portion	3	10 g	2 Weeks at 20–25^°^C	90 mL PBS Wash, no incubation required
			0.7 CFU/ test portion	10			
			2 CFU/test portion	3			
		Method A^b^ (*Aspergillus*)	0 CFU/test portion	3	10 g		*Aspergillus* enrichment broth 37 ± 1°C for 48 ± 3 h
			0.7 CFU/test portion	10			
			2 CFU/test portion	3			
		Method B^c^ (STEC/ *Salmonella*)	0 CFU/test portion	3	10 g		BPW^f^ 37 ± 1°C for 21 ± 2 h
			0.7 CFU/test portion	10			
			2 CFU/test portion	3			
		Method C^d^ (*Aspergillus*)	0 CFU/test portion	3	10 g		BPW + 0.3 g/L chloramphenicol 37 ± 1°C for 21–48 h
			0.7 CFU/test portion	10			
			2 CFU/test portion	3			
		Method D^e^ (STEC/*Salmonella*)	0 CFU/test portion	3	10 g		BPW 42 ± 2°C for 21–48 h
			0.7 CFU/test portion	10			
			2 CFU/test portion	3			

a ATCC = American Type Culture Collection (Manassas, VA).

b Method A—Gene-Up Pro *Aspergillus* (14).

c Method B—Gene-Up PRO STEC/*Salmonella* (15).

d Method C—iQ-Check *Aspergillus* (16).

e Method D—iQ-Check *Salmonella* and STEC (17,18).

f BPW = Buffered peptone water.

## Experimental

### Study Design

This method comparison study, performed by an independent third party, AOAC-certified laboratory, evaluated four proprietary assays that all utilize enrichment prior to qPCR detection of their targets and have been certified as PTMs in dried hemp/cannabis flower (14–18). These methods were compared against the PathogenDx Detect^X^ Combined assay that does not use any form of enrichment prior to tandem PCR and hybridization of the amplified targets to a DNA microarray. The methods were evaluated for the detection of *Aspergillus* spp., *Salmonella* spp., and Shiga toxin-producing *E. coli* (STEC) in dried hemp flower. Each method was evaluated according to their AOAC-validated IFU and the AOAC Appendix J validation guidance and associated standard method performance requirements for *Aspergillus*, *Salmonella*, and STEC in cannabis and cannabis products (19–21). A total of 16 samples at three levels of contamination (0 CFU/test portion, 0.7 CFU/test portion, and 2 CFU/test portion) were analyzed by each method. Results for all methods were evaluated using the POD statistical model.

### Organism Preparation and Inoculation

For inoculation of the dried hemp flower, a lyophilized culture of *A. flavus* American Type Culture Collection (ATCC) 16883, *S.* Enteritidis ATCC 13076, and *E. coli* O26 ATCC BAA-1653 was used. The lyophilized bacterial cultures were propagated on tryptic soy agar with 5% sheep blood (SBA) from a stock culture stored at −70°C. The SBA was incubated for 24 ± 2 h at 35 ± 1°C. A single colony was then transferred to brain heart infusion broth (BHI) and incubated for 24 ± 2 hours at 35 ± 1°C. The lyophilized fungal isolate was propagated in a culture flask with potato dextrose agar (PDA) from a stock culture stored at −70°C and incubated for 5–7 days at 25 ± 1°C. The culture flask was rinsed twice with 20 mL phosphate-buffered water (PBW) with 0.05% polysorbate 80.

The bacterial isolates were further diluted with BHI, and the fungal isolate with PBW. All cultures were diluted with a sterile cryoprotectant, reconstituted non-fat dry milk (NFDM), for the final dilution and freeze-dried for 48–72 h. A bulk lot of dried hemp flower was inoculated with the lyophilized culture to target the low-, intermediate-, and high-level contamination (0 CFU/test portion, 0.7 CFU/test portion, and 2 CFU/test portion). After inoculation, samples were held for 2 weeks at room temperature (20–25°C) for stabilization.

To enumerate the inoculating organisms, the lyophilized spiking suspensions were diluted in 10-fold serial dilutions and plated in duplicate on PDA. PDA was incubated at 35 ± 1°C for 48 ± 3 h. Colonies were enumerated and recorded as CFU/plate. Duplicate plates were averaged and multiplied by the dilution factor and inoculating volume to calculate the microbial population (CFU/g) of the spiking suspension.

### Confirmation Procedures

For all samples, a 1:10 dilution was created with the matrix for phosphate buffered saline (PBS) solution, PDB, and BPW. The diluted samples were incubated for 24 h for confirmation of *Salmonella* and *E. coli* O26, and 48 h for *Aspergillus* as outlined in the subsections below. Regardless of presumptive result, all samples from all methods were confirmed.

### Aspergillus

Following the 48 h of enrichment, a 10 μL aliquot of enriched sample was struck to dichloran rose bengal agar with chloramphenicol (DRBC) and PDA. Plates were incubated at 37 ± 1°C for 5–7 days. Following incubation plates were read and the presence of *Aspergillus* was confirmed via microscopic examination (19).

### Salmonella

Following incubation, 0.1 mL of primary enrichment was transferred into 10 mL Rappaport–Vassiliadis medium (RV) and 1.0 mL into 10 mL tetrathionate broth (TT). RV tubes were incubated at 42 ± 0.2°C for 24 ± 2 h in a circulating, thermostatically controlled water bath. TT tubes were incubated at 35 ± 1°C for 24 ± 2 h. Following incubation, a 10 μL aliquot of the secondary enrichments were streaked to xylose lysine deoxycholate agar (XLD) and CHROMagar^TM^ Salmonella. Plates were incubated at 35 ± 2°C for 24 ± 2 h.

Following incubation, plates were examined for growth of typical *Salmonella* colonies. A minimum of 2–3 suspect colonies from each plate were transferred to triple sugar iron agar (TSI) and lysine iron agar (LIA) slants and incubated at 35 ± 2°C for 24 ± 2 h. Following incubation, TSI and LIA slants were examined for typical reactions. Slants producing typical reactions were streaked to TSA and incubated for 35 ± 2°C for 18–24 h. Following incubation, isolates were serologically tested for both somatic O and flagellar H agglutination. Additionally, final confirmation was obtained from purified TSA isolates using the Bruker MALDI Biotyper following AOAC OMA **2017.09** (13).

#### STEC

Following enrichment, all test portions were serially diluted 1:10 in PBW. Aliquots (50 μL) of the serial dilutions were plated in duplicate onto Levine’s eosin—methylene blue agar (L-EMB) and rainbow agar (RBW) and incubated 37 ± 1°C for 18–24 h. Following incubation, plates were examined for typical colonies. Typical colonies were picked to tryptic soy agar with yeast (TSA/YE). A ColiComplete (CC) disc was placed into the heaviest area of streaking on the TSA/YE plate and incubated for 18–24 h at 37 ± 1°C.

Following incubation, the CC discs on the TSA/YE plates were observed for typical reactions (blue color change with no fluorescence under long-wave UV light) and a spot indole test was conducted. Final biochemical confirmations were obtained from a Bruker MALDI Biotyper following AOAC OMA **2017.09** (13).

Presence of *stx* was determined by performing a PTM-approved real-time screening PCR assay.

## Results

### Method Comparison

In this study we compared the performance of PathogenDx Detect^X^ Combined against four AOAC-certified qPCR methods (Table 1; 14–17). The study was designed in accordance with published *Standard Method Performance Requirements* (SMPR^®^s) for *Aspergillus*, *Salmonella*, and STEC in dried hemp flower (19–21). The goal of this method comparison study was to demonstrate that the PathogenDx Detect^X^ Combined method, an enrichment-free, end point PCR method coupled to a DNA microarray, demonstrates equivalent or superior performance to more traditional molecular methods that rely on upfront enrichment prior to qPCR detection of bacterial and/or fungal organisms. In Tables 2–4 we present POD tables comparing PathogenDx Detect^X^ Combined against the four qPCR methods. For each of the tables there are 3 uninoculated samples, 10 fractional samples, and 3 high-level samples.

**Table 2.** PathogenDx Detect^X^ Combined versus Method A and C: POD results for *Aspergillus* spp.

Matrix	Method	Contamination level/test portion (95% CI)	*n* ^a^	PathogenDx Detect^X^			Method			dPOD_C_^e^	95% CI
				*x* ^b^	POD_C_^c^	95% CI	*x*	POD_R_^d^	95% CI		
Dried hemp flower	PathogenDx Detect^X^ Combined versus Method A^g^	0	3	0	0.00	0.00, 0.56	0	0.00	0.00, 0.56	0.00	−0.56, 0.56
		1.18 (0.52, 2.45)	10	6	0.60	0.31, 0.83	6	0.60	0.31, 0.83	0.00	−0.37, 0.37
		3.07 (1.51, 11.3)	3	3	1.00	0.44, 1.00	3	1.00	0.44, 1.00	0.00	−0.56, 0.56
	PathogenDx Detect^X^ Combined versus Method C^h^	0	3	0	0.00	0.00, 0.56	0	0.00	0.00, 0.56	0.00	−0.56, 0.56
		1.18 (0.52, 2.45)	10	6	0.60	0.31, 0.83	4	0.40	0.17, 0.69	0.20	−0.20, 0.53
		3.07 (1.51, 11.3)	3	3	1.00	0.44, 1.00	3	1.00	0.44, 1.00	0.00	−0.56, 0.56

a *n* = Number of test portions.

b *x* = Number of positive test portions.

c POD_C_ = Candidate method (PathogenDx Detect^X^ Combined) confirmed positive outcomes divided by the total number of trials.

d POD_R_ = Reference method A confirmed positive outcomes divided by the total number of trials.

e dPOD_C_ = Difference between the confirmed candidate method (PathogenDx Detect^X^ Combined) result and reference method A confirmed result POD values.

f 95% CI = If the confidence interval of a dPOD does not contain zero, then the difference is statistically significant at the 5% level.

g Method A—Gene-Up Pro *Aspergillus* (14).

h Method C—iQ-Check *Aspergillus* (16).

**Table 3.** PathogenDx Detect^X^ Combined vs Method B and D—POD Results—*Salmonella* spp.

Matrix	Method	Contamination level/test portion (95% CI)	*n* ^a^	PathogenDx Detect^X^			Method			dPOD_C_^e^	95% CI
				*x* ^b^	POD_C_^c^	95% CI	*x*	POD_R_^d^	95% CI		
Dried hemp flower	PathogendDx Detect^X^ Combined versus Method B^g^	0	3	0	0.00	0.00, 0.56	0	0.00	0.00, 0.56	0.00	−0.56, 0.56
		1.18 (0.52, 2.45)	10	6	0.60	0.31, 0.83	4	0.40	0.17, 0.69	0.20	−0.20, 0.53
		2.01 (0.98, 5.43)	3	3	1.00	0.44, 1.00	3	1.00	0.44, 1.00	0.00	−0.56, 0.56
	Pathogen Dx Detect^X^ Combined versus Method D^h^	0	3	0	0.00	0.00, 0.56	0	0.00	0.00, 0.56	0.00	−0.56, 0.56
		1.18 (0.52, 2.45)	10	5	0.50	0.24, 0.76	5	0.50	0.24, 0.76	0.00	−0.37, 0.37
		2.01 (0.98, 5.43)	3	3	1.00	0.44, 1.00	3	1.00	0.44, 1.00	0.00	−0.56, 0.56

a *n* = Number of test portions.

b *x* = Number of positive test portions.

c POD_C_ = Candidate method (PathogenDx Detect^X^ Combined) confirmed positive outcomes divided by the total number of trials.

d POD_R_ = Reference method A confirmed positive outcomes divided by the total number of trials.

e dPOD_C_ = Difference between the confirmed candidate method (PathogenDx Detect^X^ Combined) result and reference method A confirmed result POD values.

f 95% CI = If the confidence interval of a dPOD does not contain zero, then the difference is statistically significant at the 5% level.

g Method B—Gene-Up PRO STEC/*Salmonella* (15).

h Method D—iQ-Check *Salmonella* and STEC (17,18).

**Table 4.** PathogenD_X_ Detect^X^ Combined versus Method B and D: POD results for STEC

Matrix	Method	Contamination level/test portion (95% CI)	*n* ^a^	PathogenDx Detect^X^			Method			dPOD_C_^e^	95% CI
				*x* ^b^	POD_C_^c^	95% CI	*x*	POD_R_^d^	95% CI		
Dried hemp flower	PathogenDx Detect^X^ Combined versus Method B^g^	0	3	0	0.00	0.00, 0.56	0	0.00	0.00, 0.56	0.00	−0.56, 0.56
		1.03 (0.41, 2.10)	10	7	0.70	0.40, 0.89	5	0.50	0.24, 0.76	0.20	−0.20, 0.53
		1.51 (0.98, 3.96)	3	3	1.00	0.44, 1.00	3	1.00	0.44, 1.00	0.00	−0.56, 0.56
	PathogenDx Detect^X^ Combined versus Method D^h^	0	3	0	0.00	0.00, 0.56	0	0.00	0.00, 0.56	0.00	−0.56, 0.56
		1.03 (0.41, 2.10)	10	5	0.50	0.24, 0.76	5	0.50	0.24, 0.76	0.00	−0.37, 0.37
		1.51 (0.98, 3.96)	3	3	1.00	0.44, 1.00	3	1.00	0.44, 1.00	0.00	−0.56, 0.56

a *n* = Number of test portions.

b *x* = Number of positive test portions.

c POD_C_ = Candidate method (PathogenDx Detect^X^ Combined) confirmed positive outcomes divided by the total number of trials.

d POD_R_ = Reference method A confirmed positive outcomes divided by the total number of trials.

e dPOD_C_ = Difference between the confirmed candidate method (PathogenDx Detect^X^ Combined) result and reference method A confirmed result POD values.

f 95% CI = If the confidence interval of a dPOD does not contain zero, then the difference is statistically significant at the 5% level.

g Method B—Gene-Up PRO STEC/*Salmonella* (15).

h Method D—iQ-Check *Salmonella* and STEC (17,18).

The POD was calculated as the number of positive outcomes divided by the total number of trials (22). In the method comparison, the POD was calculated for the PathogenDx Detect^X^ Combined method, POD_C_, each qPCR reference method, POD_R_, and the difference between Detect^X^ Combined and the qPCR reference methods, dPOD_C_ (Tables 2–4). Testing of the hemp showed no natural contamination as all of the samples produced negative results for the uninoculated samples for all of the methods tested. All methods produced fractional results at the low-level inoculation for all the pathogens evaluated. All three high-level inoculated samples for each method resulted in a positive result. The POD analysis at the fractional levels is an indication of the sensitivity of each assay. All of the assays demonstrated statistically equivalent results, POD_C_, and POD_R_, and there was no significant difference at the 5% level, 95% confidence interval (CI), indicating that each method, both with and without enrichment, provides comparable sensitivity.

### Presumptive Versus Confirmed

In the second part of the study, we confirmed the results of the presumptive methods (PathogenDx Detect^X^ Combined, Method A, Method B, Method C, and Method D) in comparison against the well-accepted confirmation methods detailed in SMPRs 2021.009, 2020.002, and 2020.012 (19–21). In Tables 5–7 we present POD tables comparing each presumptive method to the corresponding confirmation method used for each organism. For each of the tables there are 3 uninoculated samples, 10 fractional samples, and 3 high-level samples.

**Table 5.** Presumptive versus confirmed: POD results for *Aspergillus* spp.

Matrix	Method	Contamination Level/test portion (95% CI)	*n* ^a^	Presumptive			Confirmed			dPOD_CP_^e^	95% CI^f^
				*x* ^b^	POD_CP_^c^	95% CI	*x*	POD_CC_^d^	95% CI		
Dried hemp flower	PathogenDx Detect^X^ Combined	0	3	0	0.00	0.00, 0.43	0	0.00	0.00, 0.43	0.00	−0.47, 0.47
		1.18 (0.52, 2.45)	10	6	0.60	0.31, 0.83	6	0.60	0.31, 0.83	0.00	−0.25, 0.25
		3.07 (0.52, 11.3)	3	3	1.00	0.57, 1.00	3	1.00	0.57, 1.00	0.00	−0.47, 0.47
	Method A^g^	0	3	0	0.00	0.00, 0.43	0	0.00	0.00, 0.43	0.00	−0.47, 0.47
		1.18 (0.52, 2.45)	10	6	0.60	0.31, 0.83	6	0.60	0.31, 0.83	0.00	−0.25, 0.25
		3.07 (0.52, 11.3)	3	3	1.00	0.57, 1.00	3	1.00	0.57, 1.00	0.00	−0.47, 0.47
	Method C^h^	0	3	0	0.00	0.00, 0.43	0	0.00	0.00, 0.43	0.00	−0.47, 0.47
		1.18 (0.52, 2.45)	10	4	0.40	0.17, 0.69	4	0.40	0.17, 0.69	0.00	−0.25, 0.25
		3.07 (0.52, 11.3)	3	3	1.00	0.57, 1.00	3	1.00	0.57, 1.00	0.00	−0.47, 0.47

a *n* = Number of test portions.

b *x* = Number of positive test portions.

c POD_CP_ = Candidate method presumptive positive outcomes divided by the total number of trials.

d POD_CC_ = Candidate confirmed positive outcomes divided by the total number of trials.

e dPOD_CP_ = Difference between the candidate method presumptive result and candidate method confirmed result POD values.

f 95% CI = If the confidence interval of a dPOD does not contain zero, then the difference is statistically significant at the 5% level.

g Method A—Gene-Up Pro *Aspergillus* (14).

h Method C—iQ-Check *Aspergillus* (16).

**Table 6.** Presumptive vs Confirmed: POD results for *Salmonella* spp.

Matrix	Method	Contamination level/test portion (95% CI)	*n* ^a^	Presumptive			Confirmed			dPOD_CP_^e^	95% CI^f^
				*x* ^b^	POD_CP_^c^	95% CI	*x*	POD_CC_^d^	95% CI		
Dried hemp flower	PathogenDx Detect^X^ Combined	0	3	0	0.00	0.00, 0.43	0	0.00	0.00, 0.43	0.00	−0.47, 0.47
		1.18 (0.52, 2.45)	10	6	0.60	0.31, 0.83	6	0.60	0.31, 0.83	0.00	−0.25, 0.25
		2.01 (0.98, 5.43)	3	3	1.00	0.57, 1.00	3	1.00	0.57, 1.00	0.00	−0.47, 0.47
	Method B^g^	0	3	0	0.00	0.00, 0.43	0	0.00	0.00, 0.43	0.00	−0.47, 0.47
		1.18 (0.52, 2.45)	10	4	0.40	0.17, 0.69	4	0.40	0.17, 0.69	0.00	−0.25, 0.25
		2.01 (0.98, 5.43)	3	3	1.00	0.57, 1.00	3	1.00	0.57, 1.00	0.00	−0.47, 0.47
	Method D^h^	0	3	0	0.00	0.00, 0.43	0	0.00	0.00, 0.43	0.00	−0.47, 0.47
		1.18 (0.52, 2.45)	10	5	0.50	0.24, 0.76	5	0.50	0.24, 0.76	0.00	−0.25, 0.25
		2.01 (0.98, 5.43)	3	3	1.00	0.57, 1.00	3	1.00	0.57, 1.00	0.00	−0.47, 0.47

a *n* = Number of test portions.

b *x* = Number of positive test portions.

c POD_CP_ = Candidate method presumptive positive outcomes divided by the total number of trials.

d POD_CC_ = Candidate confirmed positive outcomes divided by the total number of trials.

e dPOD_CP_ = Difference between the candidate method presumptive result and candidate method confirmed result POD values.

f 95% CI = If the confidence interval of a dPOD does not contain zero, then the difference is statistically significant at the 5% level.

g Method B—Gene-Up PRO STEC/*Salmonella* (15).

h Method D—iQ-Check *Salmonella* (17).

**Table 7.** Presumptive versus confirmed: POD results for STEC

Matrix	Method	Contamination level/test portion (95% CI)	*n* ^a^	Presumptive			Confirmed			dPOD_CP_^e^	95% CI^f^
				*x* ^b^	POD_CP_^c^	95% CI	*x*	POD_CC_^d^	95% CI		
Dried hemp flower	PathogenDx Detect^X^ Combined	0	3	0	0.00	0.00, 0.43	0	0.00	0.00, 0.43	0.00	−0.47, 0.47
		1.03 (0.41, 2.10)	10	7	0.70	0.40, 0.89	7	0.70	0.40, 0.89	0.00	−0.25, 0.25
		1.51 (0.98, 3.96)	3	3	1.00	0.57, 1.00	3	1.00	0.57, 1.00	0.00	−0.47, 0.47
	Method B^g^	0	3	0	0.00	0.00, 0.43	0	0.00	0.00, 0.43	0.00	−0.47, 0.47
		1.18 (0.52, 2.45)	10	5	0.50	0.24, 0.76	5	0.50	0.24, 0.76	0.00	−0.25, 0.25
		1.51 (0.98, 3.96)	3	3	1.00	0.57, 1.00	3	1.00	0.57, 1.00	0.00	−0.47, 0.47
	Method D^h^	0	3	0	0.00	0.00, 0.43	0	0.00	0.00, 0.43	0.00	−0.47, 0.47
		1.18 (0.52, 2.45)	10	5	0.50	0.24, 0.76	5	0.50	0.24, 0.76	0.00	−0.25, 0.25
		1.51 (0.98, 3.96)	3	3	1.00	0.57, 1.00	3	1.00	0.57, 1.00	0.00	−0.47, 0.47

a *n* = Number of test portions.

b *x* = Number of positive test portions.

c POD_CP_ = Candidate method presumptive positive outcomes divided by the total number of trials.

d POD_CC_ = Candidate confirmed positive outcomes divided by the total number of trials.

e dPOD_CP_ = Difference between the candidate method presumptive result and candidate method confirmed result POD values.

f 95% CI = If the confidence interval of a dPOD does not contain zero, then the difference is statistically significant at the 5% level.

g Method B—Gene-Up PRO STEC/*Salmonella* (15).

h Method D—iQ-Check STEC (18).

Results of the presumptive versus confirmed are provided in Tables 5–7 for all assays individually. All three methods produced no results at the uninoculated level indicating that the dried hemp did not contain background pathogens. All methods produced fractional results at the low-level inoculation for all the pathogens evaluated. All three high-level inoculated samples for each method resulted in a positive result. The POD was calculated for the candidate presumptive results, POD_CP_, the candidate confirmatory results, POD_CC_, and the difference in the candidate presumptive and confirmatory results, dPOD_CP_ (Tables 5–7). The results demonstrate very good correlation between all of the presumptive methods and the confirmatory methods indicating that the methods being evaluated did not produce any false-positive or -negative results. In each of the pathogens evaluated we do observe a consistently higher sensitivity at the fractional levels for PathogenDx Detect^X^ Combined in comparison to the other qPCR methods. The POD analysis between all presumptive candidate assays and the confirmatory methods indicated that there was no significant difference at the 5% level between the number of positive results by each method.

## Discussion

The PathogenDx Detect^X^ Combined method allows the user to wash samples, collecting target pathogens, and without any enrichment, obtain results in the same day for the presence of *A. flavus, A. fumigatus, A. niger, A. terreus, Salmonella,* and a broad range of STEC. A growing concern in cannabis and food safety is how enrichment modifies the original organism makeup in the sample leading to more variable results (6–10). Enrichment followed by plating or qPCR has been the gold standard in food safety, yet these methods have not been able to prevent or mitigate large-scale outbreaks. Reports have demonstrated how enrichment can at times lead to false negatives in samples due to competition (7, 8, 11). A large concern with cannabis and food safety regulators is that without enrichment an assay is more likely to have false negatives. From this study we have demonstrated that our approach of applying a more sensitive end point PCR in combination with DNA microarrays allows for equivalent sensitivity and specificity. This mitigates enrichment bias and decreases the likelihood of false-negative results due to the utility of broad enrichment media, allowing the client to obtain a more accurate interpretation of the pathogens present in the sample being analyzed. Laboratories can be confident that by utilizing PathogenDx Detect^X^ they will obtain the same level of sensitivity and specificity, lower overall costs, and obtain results in half the amount of time preventing food spoilage.

## Conclusions

This independent laboratory method comparison study demonstrated that PathogenDx Detect^X^ Combined successfully detected *Aspergillus, Salmonella*, and STEC in dried hemp flower identifying equivalent detection of low-level positive samples in comparison to the methods evaluated (Tables 2–4). Using POD analysis, no statistically significant differences were observed between the number of presumptive positive samples detected by the PathogenDx Detect^X^ Combined assay, or the four additional assays compared in this study and the number of confirmed positives. This study demonstrates that the PathogenDx Detect^X^ Combined method is equivalent in performance to the more widely accepted methods that utilize enrichment.

## CRediT Author Statement

Benjamin A Katchman: Conceptualization, Formal Analysis, Methodology, Validation, Writing-original draft. Michael Tomchaney: Conceptualization, Methodlology, Validation. Ausitn Reuda: Methodology, Writing-review & editing. Shaun Stice: Methology, Writing-review & editing. Michael Hogan: Resources, Supervision, Writing-review & editing.
